# A High-Efficiency Fatigued Speech Feature Selection Method for Air Traffic Controllers Based on Improved Compressed Sensing

**DOI:** 10.1155/2021/2292710

**Published:** 2021-09-25

**Authors:** Yonggang Yan, Yi Mao, Zhiyuan Shen, Yitao Wei, Guozhuang Pan, Jinfu Zhu

**Affiliations:** ^1^College of Civil Aviation, Nanjing University of Aeronautics and Astronautics, Nanjing 211016, China; ^2^Air Traffic Administration Bureau, Civil Aviation Administration of China, Beijing 100022, China; ^3^State Key Laboratory of Air Traffic Management System and Technology, Nanjing 210007, China

## Abstract

Air traffic controller fatigue has recently received considerable attention from researchers because it is one of the main causes of air traffic incidents. Numerous research studies have been conducted to extract speech features related to fatigue, and their practical utilization has achieved some positive detection results. However, there are still challenges associated with the applied speech features usually being of high dimension, which leads to computational complexity and inefficient fatigue detection. This situation makes it meaningful to reduce the dimensionality and select only a few efficient features. This paper addresses these problems by proposing a high-efficiency fatigued speech selection method based on improved compressed sensing. For adapting a method to the specific field of fatigued speech, we propose an improved compressed sensing construction algorithm to decrease the reconstruction error and achieve superior sparse coding. The proposed feature selection method is then applied to optimize the high-dimension fatigued speech features based on the fractal dimension. Finally, a support vector machine classifier is applied to a series of comparative experiments using the Civil Aviation Administration of China radiotelephony corpus to demonstrate that the proposed method provides a significant improvement in the precision of fatigue detection compared with current state-of-the-art approaches.

## 1. Introduction

IATA (the International Air Transport Association) has predicted that China will become the largest civil aviation market in the world by around 2025, with China's civil aviation involving the flow of 1.6 billion passengers by around 2037 [1]. The rapid development of civil aviation represents the great challenge to air traffic control and contributes to increasing shortages of air traffic controllers (ATCs). The resulting high workloads can increase the fatigue experienced by ATCs, thus increasing the probability of human error and the associated dangerous consequences for aviation safety [2]. Research studies have demonstrated that greater fatigue is closely associated with higher risk [3]. This situation has resulted in considerable attention being paid to the accurate detection of fatigue in ATCs among researchers in the field of civil aviation.

Fatigue in ATCs can be measured using a multitude of methods and tools, which can be grouped into two categories: subjective and objective methods [4]. Subjective self-rating scales and questionnaires have been the most-important sources of data for assessing both ATC and pilot fatigue [5, 6]. Two renowned and validated subjective fatigue/sleepiness scales are the Karolinska sleepiness scale [7] and NASA's task load index [8]. Although subjective methods are easy to implement, they perform poorly in detecting a fatigue state rapidly, including real time. Therefore, objective methods have received a considerable amount of research interest. There are two categories of popular objective methods based on their different manifestations: (1) methods based on physiological parameters, including heart rate, blood pressure, breathing rate, electroencephalogram, and skin electricity [9–11], and (2) methods that directly record observable body actions, including voice strength, eye movement, blink times, yawning, and nodding frequency [12]. These objective methods are more accurate and can be used to formulate a reliable physiological fatigue index. The main disadvantage of these monitoring techniques is that their intrusiveness usually results in aversion and disturbance to the ATC, which will reduce their accuracy.

The rapid developments in speech recognition have resulted in vocal feature-based methods recently emerging as the preferred avenue for research into fatigue in ATCs [13]. Vocal features are convenient to collect and analyse, given that the main job of ATCs involves communicating with pilots via radiotelephony, and regulations specify that all voice records must be preserved for a certain period of time. There are several analyses in the literature for the connection between vocal features and fatigue [14, 15]. In 2006, Greeley et al. demonstrated that voice features show strong correlations with fatigue in the sleep onset latency test [16]. Krajewski introduced a fatigue eigenvector composed of linear speech features such as the fundamental frequency, resonance peak, and mel-frequency cepstrum coefficient (MFCC) [17]. However, the reported average accuracy when using these features was 76.5%, which is inadequate for the work performed by ATCs.

It has been demonstrated that the detection accuracy of fatigued speech is greatly affected by feature extraction and efficient features' selection [15]. It has recently become convenient to extract common speech features such as pitch, energy, and MFCC using commercial software (e.g., Opensmile) [18]. In addition, some state-of-the-art approaches utilizing nonlinear features based on wavelet decomposition and the fractal dimension [19] have shown more efficient results in detecting ATC fatigue. Overflow features result in a difficult trade-off between computational complexity and accuracy. Furthermore, the duplicated features obtained by different methods will confuse the subsequent recognition network, which consequently leads to inefficient results in detecting fatigue [20]. This situation indicates the need to achieve efficient features' selection and reduce the dimensionality of features.

Compressed sensing (CS) is a sub-Nyquist sampling technique that allows a sparse signal to be reconstructed reliably from a set of measurements to reduce the signal redundancy and reconstruction costs [21]. Many researchers have attempted to utilize this characteristic in exploring the performance of CS in dimension reduction and feature selection. For example, Haneche et al. proposed a novel speech enhancement approach based on the CS framework in 2019 [22], while Langari et al. extracted the best subset of features for speech emotion recognition by combining with CS in 2020 [23]. Although the technique of CS is beneficial for speech recognition, a considerable challenge is determining a well-designed measurement matrix that accurately represents the corresponding specific target speech signal. For this reason, the goal of this paper is to improve the conventional framework of CS to achieve the feature selection of speech, which will lead to a higher fatigue detection rate for ATCs using a popular machine learning training network, such as a support vector machine (SVM).

The rest of this paper is organized as follows.  Section 2 briefly introduces the basic theory of CS, Section 3 proposes a fatigued speech detection network and describes an improved CS construction algorithm (ICSCA) in detail.  Section 4 reports on the series of experiments performed to test our new method and conclusions are drawn in Section 5. And, all the terminologies used in this paper are illustrated in Table 1.

## 2. Compressed Sensing

CS was proposed by Candes and Donoho, who constructed the initial theoretical framework consisting of signal sparse coding, measurement matrix construction, and a reconstruction algorithm. In brief, CS can achieve complete sampling to the original signal at a sampling rate that is much lower than the Nyquist sampling theorem and reconstruct the original signal using only a small proportion of the sampled data. The detailed description is shown in Figure 1.

In Figure 1, *XϵR*^*N*^ denotes the original signal and *YϵR*^*M*^ is the final compressed signal, and *M* is usually smaller than *N*. In addition, Ψ*ϵR*^*N∗N*^ and Φ*ϵR*^*M∗N*^ indicate the sparse matrix and measurement matrix, respectively.

### 2.1. Sparse Coding

CS theory is based on the assumption that the signal is sparse or highly compressible; in other words, most of the signal values are either zero or small enough to be ignored. Even though the signals under consideration often do not satisfy the sparse condition, it might be possible to find a basic matrix to transform the original signal linearly and ensure that the coefficient vector is sparse, in case of which the original signal also exhibits sparsity. The formula for sparse coding is as follows:

(1) $$\begin{array}{c} x=\Psi S, \end{array}$$

where S*ϵR*^*N*^ represents the coefficient vector, and only *K* of the *N* signal entries are nonzero (*K* ≪ *N*). The selection of the sparse matrix depends on the inherent characteristics of the signal. The common methods used in the sparse representation include the curvelet transform, wavelet transform, barren transform, discrete cosine transform, and discrete Fourier transform.

### 2.2. Selection of Measurement Matrix

Another major problem in CS is how to choose measurement matrix Φ. For a sparse one-dimensional signal, a measurement matrix Φ is constructed to compress the original signal and obtain a measurement signal, which can be expressed as follows:

(2) $$\begin{array}{c} y=\Phi \Psi S, \end{array}$$

where *A*=ΦΨ*εR*^*M∗N*^ is defined as the sensing matrix. Generally, the restricted isometry property (RIP) defined in Definition 1 is the property that sensing matrix *A* needs to satisfy.

**Definition 1 .**

For any sparse signal *x* and measurement matrix Φ, there exists *δ*_*k*_ ∈ (0,1), and *δ*_*k*_ is the minimum value satisfying equation (3); then, it is called *δ*_*k*_, the rip constant of order *k*  of Φ:

(3) $$\begin{array}{c} \left(1-\delta_{k}\right){\left\|x\right\|}_{2}^{2}\leq {\left\|\Phi x\right\|}_{2}^{2}\leq \left(1+\delta_{k}\right){\left\|x\right\|}_{2}^{2}. \end{array}$$

The purpose of the RIP is to ensure that the “redundant” information discarded in the process of compression measurement is controlled within an acceptable range and to prevent useful information from being discarded. The RIP has been proved to be a sufficient condition for the existence of a single feasible solution of equation (3) [24].

### 2.3. Reconstruction Algorithm

The process of signal reconstruction is the reverse solution of equation (1). Since *M* is less than *N*, it is an NP-hard question for which it is difficult to obtain exact solutions. The signal reconstruction process is expressed as follows:

(4) $$\begin{array}{c} \underset{x}{\min,}{\left\|x\right\|}_{0},\\ s\mathrm{.t}\mathrm{.,}y=\Phi x, \end{array}$$

where ‖ ‖_0_ denotes the number of nonzero elements. In order to reduce the computational complexity, many scholars have proposed replacing the *L*_*o*_ norm with the *L*_2_ norm in order to transform the problem from nonconvex to convex. Some other algorithms have also been proposed by researchers to solve this problem, such as orthogonal matching pursuit (OMP) [25], iterative hard thresholding [26], basis pursuit [27], and compressed sampling matching pursuit [28].

In summary, when applying CS, it is necessary to ensure that the signal is sparse, which has led to some efficient reconstruction algorithms being proposed by researchers as CS theory has advanced. However, how to construct an efficient sensing or measurement dictionary for a particular type of input signal remains a challenge that needs to be overcome. Therefore, below, we propose an ICSCA that is suited to fatigued speech among ATCs.

## 3. Improved Fatigued Speech Feature Selection Method

### 3.1. Architecture of Fatigued Speech Detection

With the introduction of CS, a high-efficiency speech detection model based on the Civil Aviation Administration of China radiotelephony corpus is proposed. Some signal preprocessing methods are first applied to reduce the impact of noise added during the collection process, such as denoising, filtering, and emphasis. Wavelet decomposition is then applied to the speech signal, and the detailed coefficients of each signal layer are extracted. Inspired by a recently proposed nonlinear feature [29], the detailed fractal dimension coefficients of each signal layer are calculated to extract the ATC fatigued speech features. Furthermore, an ICSCA is applied to remove the redundant information and perform the final selection of the ATC fatigued speech feature. The accuracy of fatigue detection is calculated with the help of an SVM.  Figure 2 shows the detailed architecture of the proposed model.

### 3.2. Preprocessing and Feature Extraction

#### 3.2.1. Preprocessing

The energy of the speech signal is concentrated in the low frequency, and the high-frequency parts carry less energy. For solving this problem, the signal preemphasis is utilized to increase the high-frequency part of the speech signal, thereby to obtain the signal spectrum in the entire frequency band. The preemphasis is generally implemented by a first-order FIR high-pass digital filter and original signal *x*_*n*_ (the sample value at *n* time) can be processed as follows:

(5) $$\begin{array}{c} y_{n}=x_{n}-\mu x_{n-1}, \end{array}$$

where *y*_*n*_ is the new signal and *μ* represents the preemphasis coefficient and is set as 0.95.

The speech signal is a time-varying and unsteady process, and its characteristic parameters will change randomly over time, but in the short-term range (generally 10∼30 ms), the speech has relatively stable characteristics, that is, the speech signal has short-term stability. Therefore, if the speech signal is divided into short-term segments, then each segment can be regarded as stable. Taking the 16 K sampling frequency as an example, 256 sampling points are used as a chunk that is about 16 ms. And, the overlapping segmentation method is usually used to ensure a smooth transition between adjacent chunks. Finally, the selected stride is 64, and there are 192 sample points overlapped between two adjacent chunks.

Then, the chunk signal would be windowed due to reduction in the discontinuity of the signal at the beginning and end of the chunk. This is achieved by using the Hamming window *w*(*n*), and the final processing signal *y*_*w*_(*n*) can be obtained as follows:

(6) $$\begin{array}{c} w\left(n\right)=\left\{\begin{array}{cc} 0.54-0.46\left[\frac{2\pi n}{N-1}\right], & 0\leq n\leq N-1,\\ 0, & \text{other condition,} \end{array}\right. \end{array}$$

(7) $$\begin{array}{c} y_{w}\left(n\right)=y\left(n\right)\times w\left(n\right). \end{array}$$

Based on the former signal preprocess, the two typical and prevalent speech features (pH [30] and SWFF [31]) were selected to verify our proposed methods better, which are based on the speech linear and nonlinear research theory separately. The basic signal process of these two methods is introduced in the follow sections.

#### 3.2.2. pH Vocal Source Feature

The pH is a time-frequency feature used in a speaker recognition and verification system [30]. Research shows that this feature is closely related to the excitation source and consists of a vector containing the Hurst index [32]. Then, the Hurst exponent (0 < *H* < 1) expresses the time correlation or scaling degree of the speech signal. Its autocorrelation coefficient function (ACF) decays gradually in the following form:

(8) $$\begin{array}{c} \rho \left(k\right)∼H\left(2H-1\right)k^{2\left(H-2\right)},\;k⟶\infty , \end{array}$$

where the value of *H* can be associated with the spectral characteristics of {*X*(*i*)}_*i*=1_^*N*^. The detailed extraction process can be shown in Figure 3 [30].

  Step 1: the discrete wavelet transform (DWT) is applied to decompose speech signals into approximate coefficients (*a*(*l*, *k*)) and detail coefficients (*d*(*l*, *k*)). *l* is the decomposition scale (*l*=1,2,…, *J*) and *k* is the coefficient index of each scale.
  Step 2: for each scale *l*, variance *σ*_*l*_^2^=(1/*n*_*l*_)∑_*k*_*d*(*l*, *k*)^2^ is derived from the detail coefficient, where *n*_*l*_ is the number of possible coefficient values of each scale. The value of *H* is obtained as *H*=(1+*α*)/2.
  Step 3: the pH is composed of *l*+1 values in *H*[*H*_0_, *H*_1_, *H*_2_...*H*_*l*_], and component *H*_0_ is calculated from the original speech signal. Other values [*H*_0_, *H*_1_, *H*_2_ … *H*_*l*_] are obtained by repeating Steps 1 to 2 for each *l* detail coefficients' sequence.

#### 3.2.3. Speech Wavelet Fractal Feature (SWFF)

The theory of fractal dimension (FD) and wavelet decomposition are applied in extracting SWFF feature. Fractal is a complex system whose complexity can be described by a noninteger dimension called the fractal dimension (FD). It can be defined by data and calculated approximately and experimentally. It is related to *H* as follows [33]:

(9) $$\begin{array}{c} H=2-D, \end{array}$$

(10) $$\begin{array}{c} D=\underset{\varepsilon ⟶0}{\lim}\left[\frac{\log\;N\left(\varepsilon \right)}{\log\left(1/\varepsilon \right)}\right], \end{array}$$

where *D* represents the fractal dimension, *ε* is the side length of a small cube, and *N*(*ε*) is the number needed to cover the measured geometry with the small cube.

In the process of wavelet decomposition, inspired by [31], the Daubechies wavelet was chosen as the wavelet basis function because it is highly consistent with our requirements. And, the frequency distribution of speech signals on each scale after wavelet decomposition is shown in Figure 4, where high-frequency coefficient is the detail coefficient.

Then, the detailed calculation of FD can be introduced as follows:

Step 1: a time series {*X*(*i*)}_*i*=1_^*N*^ with length *N* is set up. There are *k* new time series *X*_*k*_^*m*^ that are obtained by reconstructing the time series with a delay method.
Step 2: the curve length *L*_*m*_(*k*) of each *X*_*k*_^*m*^ can be calculated using the following formula:
  (11) $$\begin{array}{c} L_{m}\left(k\right)=\frac{1}{k}\left[\left(\sum_{i=1}^{\mathrm{int}\left(N-m/k\right)}\left|X\left(m+ik\right)-X\left(m+\left(i-1\right)k\right)\right|\right)\times \frac{N-1}{\mathrm{int}\left(N-m/k\right)k}\right]. \end{array}$$
Step 3: the length of the total sequence can be approximated as the average of the length of the sequence curve generated by *k* delays. For different values of *k*, a set of curve data related to *k* and *L* (*k*) can be obtained.

In the end, the detailed SWFF feature can be obtained from the following formula:

(12) $$\begin{array}{c} D\left(d_{i}\right)=\text{FD}\left[d_{i},k_{\max}\left(d_{i}\right)\right]\;i=1,2,3,4, \end{array}$$

(13) $$\begin{array}{c} \text{SWFF}=\left[D\left(x\right),D\left(d_{1}\right),\ldots D\left(d_{4}\right)\right], \end{array}$$

where FD refers the FD calculation method and *k*_max_ is set as 10. *D*(*d*_*i*_) represents the FD of the detail coefficients of *i*^th^ layer.

### 3.3. Improved CS Construction Algorithm

The sensing dictionary and measurement matrix are constructed based on the modified *t*-mean index. The inner product of *ϕ*_*i*_ and *ε*_*i*_ is made equal to 1, such as in equation (6), which defines the *t*-mean coherence coefficient as

(14) $$\begin{array}{c} \mu_{t}\left(\Phi \right)≜\frac{\sum_{1\leq i,j\leq N,i\neq j}\left(\left|G\left(i,j\right)\right|\geq t\right)\left|G\left(i,j\right)\right|}{\sum_{1\leq i,j\leq N,i\neq j}\left(\left|G\left(i,j\right)\right|\geq t\right)|}, \end{array}$$

where *G*(*i*, *j*) represents the element in row *i* and column *j* of the Gram matrix. The absolute coherence coefficient is the average value of all nondiagonal elements whose absolute values in the Gram matrix exceed a certain threshold *t*. A greedy algorithm is then used to make the Gram matrix closer to the ideal Gram matrix. Specifically, the nondiagonal elements are gradually reduced to near 0. Finally, Φ and Ψ can be constructed when *μ*_*t*_(Φ, Ψ) satisfies the threshold.

The above process can be described as follows:

(15) $$\begin{array}{c} \underset{\Phi ,\Psi }{\arg\min}{\left\|\Psi^{T}\Phi -I\right\|}_{F}^{2}. \end{array}$$

The value of threshold *t* can be set to *t* > 0 to reduce the number of iterations because matrix *G*′ cannot be completely iterated into *I*, and the nondiagonal elements in *G*′ cannot be made equal to zero. It is proved that the minimum value of nondiagonal elements in the ETF (wqual-dimensional tight frame) matrix is

(16) $$\begin{array}{c} t_{E}=\pm \sqrt{\frac{n-m}{m\left(n-1\right)}}. \end{array}$$

The construction process and characteristics of *G*′ are very similar to the ETF matrix. In this case, equation (12) can be modified as

(17) $$\begin{array}{c} \underset{\Phi ,\Psi }{\arg\min}{\left\|\Psi^{T}\Phi -H\right\|}_{F}^{2}, \end{array}$$

where *H* ∈ *R*^*N∗N*^, the diagonal element of matrix *H* is equal to 1, and nondiagonal elements are equal to *t*_*E*_*∗*sign(*G*′(*i*, *j*)).

Solving equation (14) yields the measurement matrix and sensing dictionary. Equation (14) can be decomposed into the following two problems that are solved iteratively:

(18) $$\begin{array}{c} \text{Problem }\left(1\right):\;\Phi =\underset{\Phi }{\arg\min}{\left\|\Phi^{T}\Phi -H\right\|}_{F}^{2}, \end{array}$$

(19) $$\begin{array}{c} \text{Problem }\left(2\right):\;\Psi =\underset{\Psi }{\arg\min}{\left\|\Psi^{T}\Phi -H\right\|}_{F}^{2}. \end{array}$$

Evaluation and performance assessment are calculated iteratively by using OMP and equation (11). If the difference between the results of successive iterations is less than the threshold or the number of iterations exceeds the set maximum number of iterations, the algorithm is terminated.

The gradient method is used to solve Problem (1). The values of the nondiagonal elements of the matrix can be reduced to reduce the coherence between different columns. The optimization process is described as follows:

Step 1: define the cost function as **C**=‖Φ^**T**^Φ − *H*‖_**F**_^2^.
Step 2: calculate the gradient of the cost function:
  (20) $$\begin{array}{c} \frac{\partial C}{\partial \Phi }=\frac{\partial }{\partial \Phi }\text{Tr}\left\{{\left(\Phi^{T}\Phi -H\right)}^{T}\left(\Phi^{T}\Phi -H\right)\right\}. \end{array}$$
Simplify this to
  (21) $$\begin{array}{c} \frac{\partial C}{\partial \Phi }=4\Phi \left(\Phi^{T}\Phi -H\right). \end{array}$$
Step 3: the complete iteration equation is
  (22) $$\begin{array}{c} \Phi_{\left(k+1\right)}=\Phi_{\left(k\right)}-\beta \frac{\partial C}{\partial \Phi_{k}}, \end{array}$$
where *k* is the number of iterations and *β* is the step size, which is set as 0.001.
Step 4: use OMP to evaluate the coherence coefficient of *t* and evaluate whether the difference between the results of two successive iterations is less than the threshold.

Two points need to be considered when solving Problem (2): (i) ensuring the correlation between the sensing dictionary and measurement matrix throughout the process and (ii) ensuring the consistency between Ψ and Φ, where *μ*_*t*_(Ψ, Φ) should be as small as possible. For overcoming the former difficulty, we propose methods as follows.

Matrix *G*′=Ψ^*T*^Φ is first constructed. Then, using the taut operator to shrink the nondiagonal elements in the matrix, approximation degree *H* is gradually reduced. Finally, a pair of perceptual dictionaries and measurement matrices can be obtained by singular value decomposition.

The value range of the nondiagonal elements of the matrix is [1, −1] because matrix Ψ and matrix Φ are initially column normalized. Applying the tighten operator further narrows this range to [−*γ*, *γ*], where *γ* < 1. A simple and easy-to-implement operator is proposed for mapping from [1, −1] to [−*γ*, *γ*]:

(23) $$\begin{array}{c} \rho =\frac{4}{\pi }*\gamma *\;\arctan\left(G^{\prime }\left(i,j\right)\right). \end{array}$$

It can be seen that the above tightening operator can adjust the range of matrix *G*′ nondiagonal elements in iterations with only one parameter, *γ*, which is set as 0.4.

Utilizing the SVD decomposition yields

(24) $$\begin{array}{c} G^{\prime }=U^{T}VW. \end{array}$$

The diagonal elements in matrix *V* are nonnegative, and all diagonal elements are arranged from the upper-left corner to the lower-right corner. In order to be closer to *H*, set the maximum *M* elements in *V*_*M*_ to be retained and then construct as follows:

(25) $$\begin{array}{c} \Psi =V_{M}^{1/2}U,\\ \Phi =V_{M}^{1/2}W. \end{array}$$

At the same time, in order to ensure that the inner product of corresponding atoms is 1, it should be treated according to the following formula:

(26) $$\begin{array}{c} \phi_{i}=\frac{\phi_{i}}{{\left\|\phi_{i}\right\|}_{2}},\\ \varepsilon_{i}=\frac{\varepsilon_{i}}{\left|\langle \varepsilon_{i},\phi_{i}\rangle \right|}. \end{array}$$

Above all, we construct a pair of sensing dictionary Ψ and measurement matrix Φ with a weak cross correlation.

### 3.4. SVM Settings

An SVM is a classification model whose mathematical strategy involves maximizing the interval of different kinds of data. Therefore, an SVM can be formalized as a convex quadratic programming problem. Here, a WLS-SVM (weighted-least-squares SVM) [34] is used for the classification process, which is formulated as

(27) $$\begin{array}{c} {\hat{y}}_{v}=\frac{\sum_{i=1}^{C}P_{iv}{\hat{y}}_{iv}}{\sum_{i=1}^{C}P_{iv}}. \end{array}$$

The *i*^th^ weighting coefficient of *x*_*v*_ is calculated as

(28) $$\begin{array}{c} P_{iv}\left(x_{iv}\right)=A_{iv}^{1}\left(x_{iv}^{1}\right)A_{iv}^{2}\left(x_{iv}^{2}\right)\cdots A_{iv}^{n}\left(x_{iv}^{n}\right), \end{array}$$

(29) $$\begin{array}{c} A_{ij}^{t}=\exp\left(-\left(\frac{x_{ij}-\theta_{i}^{t}}{\beta_{i}^{t}}\right)\right),\theta_{i}^{t}=z_{i}^{t}, \end{array}$$

(30) $$\begin{array}{c} \beta_{i}^{t}=\lambda \sqrt{\frac{\sum_{j=1}^{N}{\left(\mu_{ij}\right)}^{m}{\left(x_{ij}^{t}-\theta_{i}^{t}\right)}^{2}}{\sum_{j=1}^{N}{\left(\mu_{ij}\right)}^{m}}}, \end{array}$$

where *A*_*ij*_^*t*^ represents the membership grade, *t*=1,2,…, *n*. The WLS-SVM utilizes fuzzy *c*-means clustering methods to decide the rule number, which is based on the following formula:

(31) $$\begin{array}{c} \min J_{m}\left(\mu_{ij},z_{i}\right)=\overset{C}{\underset{i=1}{\sum }}\overset{N}{\underset{j=1}{\sum }}{\left(\mu_{ij}\right)}^{m}x_{j}-z_{i}{}^{2}, \end{array}$$

(32) $$\begin{array}{c} \sum_{i=1}^{C}\mu_{ij}=1;\;0<\overset{N}{\underset{j=1}{\sum }}\mu_{ij}<N, \end{array}$$

where *m* ∈ (1, *∞*) denotes a fuzzy exponent, *μ*_*ij*_(*μ*_*ij*_ ∈ *U*) is the degree to which *x*_*j*_ belongs to the *i*^th^ rule, and *z*_*i*_ is the *i*^th^ cluster center. The advantage of a WLS-SVM is that general errors including noise in the input and output variables are considered as empirical errors.

Furthermore, in terms of the selection of the Gauss kernel function, we finally use the radial basis function (RBF) due to its superior antijamming ability for noise in data. The RBF kernel in this research is the same as the activation function used by Mu et al. [35]. The mathematical model of the kernel function is as follows:

(33) $$\begin{array}{c} K\left(x_{i},x_{j}\right)=\exp\left(-\gamma x_{i}-x_{j}{}^{2}\right),\;\gamma >0, \end{array}$$

where *γ* is the parameters of the kernel function.

## 4. Experimental Results

Experimental results were obtained on a Windows 10 personal computer equipped with a 64 bit Intel Core i5-9300H CPU running at 2.4 GHz and with 8 GB of RAM. All of the proposed methods were implemented using Python (version 3.7) and TensorFlow (version 1.14.0) software.

### 4.1. Datasets and Parameters

A fatigued speech dataset [31] consisting of 1606 speech samples from ATC radiotelephony was used in the experiment depicted in Table 2. Due to the proportion of samples representing fatigued speech being less than for normal speech samples, we finally selected 824 speech samples from the dataset (412 fatigued speech samples and 412 normal speech samples) to ensure the authority of experimental results.

The SWFF was then extracted as the original signal feature. The dimension of the SWFF was 256, and according to the progress of CS, we set the final feature dimension to be 32.

During the set of the SVM, the 824 speech samples were divided into *K* = 6 groups (the overall average). Each subset dataset was used as a verification set, and the remaining subset dataset was used as a training set so that *K* models could be obtained. The average classification accuracy of the final verification set of these *K* models was used as the performance index of the classifier under this K-CV. The penalty factor was set to *c*=9.7656 × 10^−4^, and the gamma parameter was *γ* = 0.5.

### 4.2. Results and Analysis

In this section, the experiments were conducted by using two types of prevalent fatigue features (PH and SWFF). And, the sparse autoencoder (SAE) [36] was utilized to replace the SVM classifier. Furthermore, the Gauss random matrix and uncompressed sample were selected for comparisons with the ICSCA. The fatigue state detection results obtained by using these two nonstop measurement matrix construction algorithms for feature sampling are shown in Figures 5 –7 and Table 3.

Overall, it was clear that SWFF feature played better detection performance with the same classification methods. Considering the use of different classifiers, we can see that the SAE method consumed less time, but the average accuracy was far lower than the SVM.

In terms of the function of different measurement matrices, compared with the detection results without feature sampling, the accuracy of ATC fatigue state detection for Gaussian random matrix algorithm feature sampling was reduced by about 2%, while the detection results with proposed ICSCA were improved to 85.11% (pH) and 94.25% (SWFF) separately. Finally, it can see that the proposed ICSCA method also has the fastest operation speed of 1.37 minutes (pH) and 1.21 minutes (SWFF), which features the highest accuracy rate of 97.11%, when compared with DDL is 93.10%, while pH is 60.36% and SWFF is 71.39%. These findings demonstrated that the ICSCA proposed in this study provides better improvement in both detection accuracy and operation time.

## 5. Conclusions

In order to quantitatively and fast detect fatigue condition of ATCs, we proposed a CS-based framework for detecting fatigue from speech of ATCs. Then, an improved compressed sensing reconstruction algorithm is proposed to decrease the reconstruction error and achieve superior sparse coding, which was applied to fatigued speech selection with redundant information in the original feature vector removed. Finally, pH and SWFF speech features are applied to a series of comparative experiments using the Civil Aviation Administration of China radiotelephony corpus to demonstrate that the proposed method provides a significant improvement in the precision of fatigue detection compared with current state-of-the-art approaches.

## Figures and Tables

**Figure 1:** Flowchart of compressive sensing.

**Figure 2:** Architecture of fatigued speech detection.

**Figure 3:** An example of the pH estimation, considering *l*=2 decomposition stages.

**Figure 4:** Frequency distribution of speech signal on different scales after wavelet decomposition.

**Figure 5:** The average accuracy with Gaussian random matrix. (a) pH feature; (b) SWFF feature.

**Figure 6:** The average accuracy with uncompressed sampling. (a) pH feature; (b) SWFF feature.

**Figure 7:** The average accuracy with proposed ICSCA. (a) pH feature; (b) SWFF feature.

**Table 1:** List of terminologies used in this paper.

ATC	Air traffic controller
ATCs	Air traffic controllers
MFCC	Mel-frequency cepstrum coefficient
CS	Compressed sensing
ETF	Equal-dimensional tight frame
FD	Fractal dimension
ICSCA	Improved CS construction algorithm (ICSCA)
NP	Nondeterministic polynomial
OMP	Orthogonal matching pursuit
RIP	Restricted isometry property
RBF	Radial basis function
SVM	Support vector machine
SWFF	Speech wavelet fractal feature
WLS-SVM	Weighted-least-squares SVM

**Table 2:** The fatigue dataset utilized in this study.

Fatigue data set	Number	Expression	Explanation
	1	Control category	*R*, area control; *A*, approach control; *T*, tower control
	2	ATC rank	5, level 5; 4, level 4; 3, level 3; 2, level 2; 1, level 1; 0, trainee
	3–10	Time (UTC)	3–6, time of starting work; 7–10, time of ending work
	11	Sex	*F*, female; *M*, male
	12 and 13	Age	Arabic numeral (age in years)
	14 and 15	Order	*Nn*, *N* is a digital indicator and *n* is an Arabic numeral indicating the *n*^th^ instruction issued by the ATC while working
	16 and 17	Status	14^th^, “-;” 15^th^, voice command; 1, error; 2, ambiguity; 3, hesitation or pause; 4, fatigue

**Table 3:** Detection results based on different measurement-matrix construction methods.

Fatigue feature	Classifier	Kernel function	Measurement matrix	Average accuracy	Total time (minutes)
PH	SAE			79.67%	2.35
	SVM	RBF	Gaussian random matrix	81.61%	5.12
			Uncompressed sampling	79.36%	6.38
			**ICSCA**	**85.11%**	**1.37**

SWFF	SAE			82.86%	1.88
	SVM	RBF	Gaussian random matrix	91.52%	4.65
			Uncompressed sampling	89.31%	5.78
			**ICSCA**	**94.25%**	**1.21**

## Data Availability

The radiotelephony corpus data sampled from Air Traffic Management Bureau, Civil Aviation Administration of China, used to support the findings of this study, are available from the corresponding author upon request.

## References

[1] IATA (2018). *Forecast Predicts 8.2 Billion Air Travelers in 2037*.

[2] Irfan A., Ahmed I., Malik M. (2021). Hazards of fatigue: learning from aviation. *Bulletin of the Royal College of Surgeons of England*.

[3] Nicholas W., Bijay G., Ajay V., Lewis A., Kouhyar T. (2020). Blending human and machine: feasibility of measuring fatigue through the aviation headset. *Human factors*.

[4] Seung Young L., Kim J. K. (2018). Factors contributing to the risk of airline pilot fatigue. *Journal of Air Transport Management*.

[5] Wang X., Xu C. (2016). Driver drowsiness detection based on non-intrusive metrics considering individual specifics. *Accident Analysis & Prevention*.

[6] Lasota A. M., Hankiewicz K. (2020). Self-reported fatigue and health complaints of refuse collectors. *Central European Journal of Operations Research*.

[7] Chalder T., Berelowitz G., Pawlikowska T. (1993). Development of a fatigue scale. *Journal of Psychosomatic Research*.

[8] Riethmeister V., Bültmann U., Gordijn M., Brouwer S., Boer M. (2018). Investigating daily fatigue scores during two-week offshore day shifts. *Applied Ergonomics*.

[9] Arnau S., Möckel T., Rinkenauer G., Wascher E. (2017). The interconnection of mental fatigue and aging: an EEG study. *International Journal of Psychophysiology*.

[10] Shitong H., Jia L., Pengzhu Z., Weiqiang Z. (2018). Detection of mental fatigue state with wearable ECG devices.. *International Journal of Medical Informatics*.

[11] Hu X., Lodewijks G. (2020). Detecting fatigue in car drivers and aircraft pilots by using non-invasive measures: the value of differentiation of sleepiness and mental fatigue. *Journal of Safety Research*.

[12] Chen M.-L., Lu S.-Y., Mao I.-F. (2019). Subjective symptoms and physiological measures of fatigue in air traffic controllers. *International Journal of Industrial Ergonomics*.

[13] Nie B., Huang X., Chen Y., Li A., Zhang R., Huang J. (2017). Experimental study on visual detection for fatigue of fixed-position staff. *Applied Ergonomics*.

[14] K Anduri V. S., Emilian J., Jagadish V. (2021). *Fatigue Analysis of Vocal-Folds Using Discretized Aeroelastic Model*.

[15] Chen S., Zhao H., Chen X., Cheng F. Detecting sports fatigue from speech by support vector machine.

[16] Greeley H. P., Friets E., Wilson J. P., Raghavan S, Picone J, Berg J. Detecting fatigue from voice using speech recognition.

[17] Albornoz E. M., Sánchezgutiérrez M., Martinezlicona F., Rufiner H. Spoken Emotion Recognition Using Deep Learning.

[18] Wang C. (2020). Speech emotion recognition based on multi-feature and multi-lingual fusion. https://arxiv.org/abs/2001.05908.

[19] Ozcelikkale A. Sparse recovery with non-linear fourier features.

[20] Rodriguez-Dominguez U., Dalmau O. (2020). Hierarchical discriminative deep dictionary learning. *IEEE Access*.

[21] Chin W.-L., Kuo H.-C., Chen H.-H. (2012). Features detection assisted spectrum sensing in wireless regional area network cognitive radio systems. *IET Communications*.

[22] Haneche H., Ouahabi A., Boudr A. B. (2019). New mobile communication system design for Rayleigh environments based on compressed sensing-source coding. *Communications, IET*.

[23] Langari S., Marvi H., Zahedi M. (2020). Efficient speech emotion recognition using modified feature extraction. *Informatics in Medicine Unlocked*.

[24] Devore R. A. (2007). Deterministic constructions of compressed sensing matrices[J]. *Journal of Complexity*.

[25] Rezaiifar Y. C. P. R., Krishnaprasad P. S. Orthogonal matching pursuit: recursive function approximation with applications to wavelet decomposition.

[26] Blumensath T., Davies M. E. (2010). Normalized iterative hard thresholding: guaranteed stability and performance. *IEEE Journal of Selected Topics in Signal Processing*.

[27] Gunn R. N., Gunn S. R., Turkheimer F. E., Aston J. A. D., Cunningham V. J. (2002). Positron emission tomography compartmental models: a basis pursuit strategy for Kinetic modeling. *Journal of Cerebral Blood Flow and Metabolism*.

[28] Zhang X. W. (2012). Sparse Signal Recovery Based on Stepwise Compressed Sampling Matching Pursuit. *Signal Processing*.

[29] Wang Z., Yang C., Wei W., Yingle F. (2008). Speaker gender identification based on audio fractal dimension and pitch feature. *Journal of biomedical engineering*.

[30] Sant’Ana R., Coelho R., Alcaim A. (2006). Text-independent speaker recognition based on the Hurst parameter and the multidimensional fractional Brownian motion model. *IEEE Transactions on Audio Speech and Language Processing*.

[31] Shen Z., Pan G., Yan Y. (2020). A high-precision fatigue detecting method for air traffic controllers based on revised fractal dimension feature. *Mathematical Problems in Engineering*.

[32] Zao L., Cavalcante D., Coelho R. (2014). Time-frequency feature and AMS-GMM mask for acoustic emotion classification. *IEEE Signal Processing Letters*.

[33] Ruiz-Medina M. D., Porcu E., Fernandez-Pascual R. (2011). The Dagum and auxiliary covariance families: towards reconciling two-parameter models that separate fractal dimension and the Hurst effect. *Probabilistic Engineering Mechanics*.

[34] Sun C., Mu C., Li X. (2009). A weighted LS-SVM approach for the identification of a class of nonlinear inverse systems. *Science in China-Series F: Information Sciences*.

[35] Mu C., Zhang Y. (2019). Learning-based robust tracking control of quadrotor with time-varying and coupling uncertainties. *IEEE Transactions on Neural Networks and Learning Systems*.

[36] Shen Z., Wei Y. (2021). A high-precision feature extraction network of fatigue speech from air traffic controller radiotelephony based on improved deep learning. *ICT Express*.

